The article "The Immunomodulatory Effects of Nidus Vespae on Human Peripheral Blood Immune Cells In Vitro" was published in 2015. Journal: Evid Based Complement Alternat Med.

# The Immunomodulatory Effects of Nidus Vespae on Human Peripheral Blood Immune Cells *In Vitro*

**DOI:** 10.1155/2015/705308

**Published:** 2015-08-03

**Authors:** Ming Zhu, Yang Ling, Qiufeng Qi, Yaping Zhang, Yanqing Bao, Yongping Liu

**Affiliations:** Clinical Oncology Laboratory, Changzhou Tumor Hospital Affiliated to Soochow University, Huaide Road 44, Changzhou 213002, China

## Abstract

Nidus Vespae has been used in traditional Chinese medicine (TCM) to treat various cancers, but the underlying mechanisms were not yet clarified. This study was to investigate the effect of Nidus Vespae decoction (NVD) on tumor cell viability and immunoregulating functions of human peripheral blood immune cells. The effects on tumor cell viability, peripheral blood mononuclear cell (PBMC) proliferation activity, and the tumor cell phagocytosis of monocytes were evaluated by cell counting kit-8. Tumor-killing activity of cytotoxic T lymphocyte (CTL) was analyzed by ^51^Cr releasing assay. IgG production of B cells and cytokine (TNF-*α* and IL-6) secretion of monocytes were determined by ELISA method. Data showed that NVD has no significant inhibiting effects on gastric cancer cells growth. Nevertheless, it could obviously promote PBMC proliferation in a time- and concentration-dependent manner. After treatment with NVD, the CTL cytotoxicity against SGC-7901 was significantly greater than control. The TNF-*α* and IL-6 secretion of monocytes and the IgG production of B cells also increased remarkably. Furthermore, NVD could significantly promote the phagocytosis of monocytes on tumor cells. These results suggest that NVD appears to have an immunoenhancing effect on immune cells, indicating that Nidus Vespae is worth exploring for immunomodulatory effects in tumor treatment.

## 1. Introduction

Nidus Vespae, a traditional Chinese medicine, is the honeycomb of* Polistes olivaceus* (De Geer),* Polistes japonicus* Saussure, or* Parapolybia varia* Fabricius. It is widely distributed in China and usually harvested in autumn and winter. After removal of dead wasps, Nidus Vespae is manufactured into a traditional Chinese medicine by open-air drying. Because of the multiple pharmacological activities, including anti-inflammatory, antimicrobial, antivirus, antitumor, and anesthetic properties [1], Nidus Vespae has been used in traditional Chinese medicine (TCM) for thousands of years to treat a variety of diseases, including malignant tumors, rheumatoid arthritis, lung diseases, skin disease, digestive and urinary disorders, and dental diseases [1, 2]. Although Nidus Vespae is widely used in Chinese folk medicine, the underlying mechanisms by which it exerts therapeutic function have not been thoroughly studied, especially in antitumor therapy.

The article "The Immunomodulatory Effects of Nidus Vespae on Human Peripheral Blood Immune Cells In Vitro" was published in 2015. Journal: Evid Based Complement Alternat Med.

Cancer is considered to be one of the biggest killers of human beings all over the world. Since the cures are not yet available for most carcinomas, patients suffer from the illness and face longtime treatment. Chinese medicine inspires us to develop complementary and alternative therapy (CAM) for the treatment of cancer [3]. In recent years, several studies have been carried out to investigate the mechanisms by which Chinese medicinal herbs exert their antitumor effects. The possible mechanisms are mainly reflected in the following aspects. The first is inhibiting the growth and proliferation of tumor cells. For example, Radix Astragali (AR), which could specifically inhibit gastric cancer cells growth* in vitro* and the mechanism, is mainly cytostatic but not cytotoxic or inducing apoptosis [4]. The second is regulating the function of immune system. For instance, Bazhen decoction has been reported to be able to encourage the proliferation and activation of T lymphocytes [5].* Astragalus membranaceus*, propolis, Zingiberis rhizoma,* Ganoderma lucidum*, and so on have been shown to promote the cytokine production of immune cells [6–10]. Tenglong Buzhong decoction and Xuebijing injection reduce the count of Tregs and the levels of IL-10 and TGF-*β* in the patients of late colorectal cancer, thereby improving immune function of effector T cells [11, 12]. The third is inducing the apoptosis of tumor cells. Similar to arsenic sulfide (As4S4), the main component of realgar has been shown to induce apoptosis of gastric cancer cells both* in vitro* and* in vivo* through a p53-dependent pathway [13]. The final aspect is inhibiting the tumor angiogenesis. One example is Raddeanin A (RA), which could significantly inhibit human umbilical vein endothelial cell proliferation, motility, migration, and tube formation. RA also dramatically reduces angiogenesis in chick embryo chorioallantoic membrane, restrains the trunk angiogenesis in zebrafish, and suppresses angiogenesis and growth of human HCT-15 colorectal cancer xenograft in mice [14].

Numerous Chinese herbs appear to play an important role in the antitumor effects, especially through regulating the function of immune system. In order to explore the possible mechanisms by which Nidus Vespae extract exerts antitumor effects, extracorporeal experimental studies were carried out to investigate the influence of NVD on tumor cell viability and on the function of human peripheral blood immune cells.

## 2. Materials and Methods

### 2.1. Preparation of Nidus Vespae Decoction (NVD)

The 30 g Nidus Vespae crude drug was purchased from pharmacy of Changzhou Tumor Hospital Affiliated to Soochow University and the Nidus Vespae decoction (NVD) was prepared according to the standard of the Chinese Pharmacopeia. In brief, the Nidus Vespae was rinsed twice and soaked overnight with 1000 mL Milli-Q water (Millipore, Molsheim, France). The Nidus Vespae was decocted for 30 min after the water was boiled. The liquid was then filtered. This procedure was repeated twice. The decoctions were mixed and concentrated to approximately 25~100 mL by heating. After centrifuging for 10 min at 3000 rpm, the residue was discarded and about 43 mL NVD was collected. The drug concentration was calculated to be 700 mg/mL. Then, part of the concentrated NVD was taken for LPS detection and the remaining was packed and stored at −80°C for later use. The LPS content in NVD was detected by Limulus Amebocyte Lysate (LAL) test according to the manuscript of ToxinSensor Gel Clot Endotoxin Assay Kit (GenScript, Nanjing, China). The result showed that the LPS concentration in the concentrated NVD was between 2.5 and 5 EU/mL, as the working concentration of NVD in this essay was less than or equal to 10000 *μ*g/mL, with the LPS concentration approximately at most 0.071 EU/mL, which was lower than the negative reference value of this kit (0.25 EU/mL). Therefore, the Nidus Vespae decoction we prepared was suitable for our experiment.

The article "The Immunomodulatory Effects of Nidus Vespae on Human Peripheral Blood Immune Cells In Vitro" was published in 2015. Journal: Evid Based Complement Alternat Med.

### 2.2. Analysis of Tumor Cell Viability

Human gastric cancer cell lines SGC-7901, HGC-27, and NCI-N87 were obtained from the cell bank of the Shanghai Institutes for Biological Sciences, Chinese Academy of Sciences. Cells were maintained in RPMI 1640 medium (Hyclone Laboratories, USA), supplemented with 10% fetal bovine serum (Hyclone Laboratories, USA), and incubated at 37°C in 5% CO_2_ humidified air. The cell concentration was adjusted to 1 × 10^6^/mL, seeded into a 96-well plate with 100 *μ*L a well, and cultured with 100 *μ*L NVD at final concentration of 10000, 5000, 2500, 1000, 100, and 10 *μ*g/mL for 24 h. The plate was centrifuged at approximately 800 ×g for 5 minutes and then the supernatant was discarded. Then, 100 *μ*L RPMI 1640 containing 10% CCK-8 was added to each well to detect the absorbance (*A*) with a microplate reader (BIO-RAD, USA) at 490 nm. The blank control wells were used for zeroing absorbance. For each experiment, 10 wells containing drug-free medium were allocated as the control. Tumor cell viability was calculated using the background corrected absorbance by the following formula: tumor cell viability (%) = *A* experimental well/*A* untreated control well × 100%, where *A* is absorbance.

### 2.3. Assessment of PBMC Proliferation Ability

Heparinized venous blood was obtained from 5 gastric cancer patients after approval by the Ethics Committee. Peripheral blood mononuclear cells (PBMCs) were isolated with Ficoll cell isolation reagent (Sigma Chemical Co., USA). Briefly, 5 mL of heparinized blood was mixed with an equal volume of RPMI-1640 medium. Samples were layered over 5 mL Ficoll-Histopaque in a 15 mL plastic centrifuge tube. After centrifuging at 2500 rpm for 30 min at room temperature, the interface layer of PBMC was carefully sucked out and washed twice with RPMI-1640 medium at 1500 rpm for 10 min.

The article "The Immunomodulatory Effects of Nidus Vespae on Human Peripheral Blood Immune Cells In Vitro" was published in 2015. Journal: Evid Based Complement Alternat Med.

The PBMC was resuspended in culture medium at a concentration of 1 × 10^6^/mL and added into a 96-well plate, with 100 *μ*L a well. Next, according to the experimental design, 100 *μ*L ConA at a final concentration of 5 *μ*g/mL or NVD at different concentrations was added to each well (equal volume of medium for negative control). Three identical plates were set according to the above description and incubated at 37°C for 24, 48, and 72 hours, respectively. Afterwards, the plates were centrifuged at approximately 800 ×g for 5 minutes. The supernatant was discarded. And then, 100 *μ*L RPMI 1640 containing 10% CCK-8 was added into each well to detect the OD values and to calculate the PBMC proliferation rate.

### 2.4. Determination of CTL Activity

Mitomycin C treated gastric cancer cell line SGC-7901 (1 × 10^5^) and PBMC (2 × 10^6^) were cultured with 2500 *μ*g/mL NVD (with PBS as control) for 5 days to induce cytotoxic T lymphocyte (CTL) responses specific for SGC-7901. The tumor-killing activity of CTL was assessed by ^51^Cr releasing assay. SGC-7901 (1 × 10^4^) was seeded onto fibronectin-pretreated (50 *μ*L/well at 10 *μ*g/mL) 96-well microplates and loaded overnight with ^51^Cr (1 *μ*Ci/mL). After washing, CTLs were added to the ^51^Cr-labelled SGC-7901 target cells in effector/target ratios of 10 : 1, 20 : 1, and 40 : 1. After 16 h of coculture, counts per min (cpm) radioactivity was determined and cytotoxicity index (%) was calculated by the following formula: cytotoxicity index (%) = [(*a* − *b*)/(*c* − *b*)] × 100%, where *a* is the cpm released from target cells incubated with CTLs, *b* is the cpm released spontaneously from target cells incubated alone, and *c* is maximal cpm released from target cells incubated with 1% Nonidet P-40.

### 2.5. Analysis of IgG Production

PBMCs (5 × 10^5^/well) were treated with 0.005% SAC or NVD at different concentration levels (5000, 2500, and 250 *μ*g/mL) in a 24-well plate for 24 h at 37°C and 5% CO_2_. Afterwards, the supernatant was harvested for the measurement of IgG production using enzyme linked immunosorbent assay (ELISA), according to manufacturer's protocol (eBioscience, USA). Briefly, a Corning Costar 9018 (Corning, USA) was coated with 100 *μ*L/well of capture antibody specific to IgG. The plate was washed and blocked before 100 *μ*L of the supernatants and serially diluted specific standards were added to the respective wells. Following a series of washing, the captured IgG was detected using the specific conjugated detection antibody. The substrate reagent was added into each well. After color development, the plate was read at 450 nm, using a microplate reader.

The article "The Immunomodulatory Effects of Nidus Vespae on Human Peripheral Blood Immune Cells In Vitro" was published in 2015. Journal: Evid Based Complement Alternat Med.

### 2.6. Determination of Cytokine Production by Monocytes

The PBMC isolated from 20 mL heparinized blood was incubated in 25 cm^2^ culture bottle at 37°C with 5% CO_2_ for 2 h. Next, nonadherent cells were removed and human adherent monocytes were collected with a cell scraper (NEST, China). Monocytes (5 × 10^5^/well) were treated with LPS at 5 *μ*g/mL or NVD at different concentrations (5000, 2500, and 250 *μ*g/mL) in a 24-well plate for 24 h at 37°C and 5% CO_2_. Afterwards, the supernatant was harvested for the measurement of cytokines (TNF-*α* and IL-6) using enzyme linked immunosorbent assay (ELISA), according to manufacturer's protocol (eBioscience, USA).

### 2.7. Analysis on Tumor Cell Phagocytosis of Monocytes

Monocytes (2 × 10^5^/well, with complete medium as control) were treated with 2500 *μ*g/mL NVD (with PBS as control) in a 96-well plate. After 24 hours, 1 × 10^4^ gastric tumor cells SGC-7901 (with complete medium as control) were added and cultured for 48 h. The plate was centrifuged at approximately 800 ×g for 5 minutes; then the supernatant was discarded. And then, 100 *μ*L RPMI 1640 containing 10% CCK-8 was added, respectively, to detect the OD values.

### 2.8. Statistical Analysis

Statistical significance was calculated using GraphPad Prism (GraphPad Software Inc., San Diego, CA, USA) and the data were presented as mean ± SD. Tumor cell viability, IgG production, cytokine levels, and phagocytosis of monocytes were analysed by one-way ANOVA. Two-way ANOVA with a Bonferroni posttest was used to analyse the PBMC proliferation and tumor cell-killing activity of CTL. All statistical methods have been stated in figures. *P* values < 0.05 were considered statistically significant.

## 3. Results

### 3.1. Effects of NVD on Tumor Cells Viability

The cytotoxicity of NVD on gastric tumor cells was tested by cell counting kit-8. There were no significant differences between all concentrations, although increased tendencies of viability were observed in Figure 1. It indicates that NVD does not lead to the SGC-7901, HGC-27, and NCI-N87 toxicities in the studied concentrations (10~10000 *μ*g/mL).

### 3.2. Effects of NVD on PBMC Proliferation Ability

PBMC were incubated with and without NVD at different concentrations. In order to find the optimal concentration of NVD, it was tested at seven concentration levels of 75, 150, 300, 600, 1250, 2500, and 5000 *μ*g/mL at 24 h, 48 h, and 72 h. Compared to the PBS control groups, PBMC promotion was observed very significantly (*P* < 0.0001) at NVD concentration levels of 600, 1250, 2500, and 5000 *μ*g/mL and to a lesser extent (*P* < 0.001) at 150 and 300 *μ*g/mL. The lowest concentration of NVD (75 *μ*g/mL) did not show any promotion. Furthermore, the promotion of NVD on PBMC proliferation displayed significant time-dependence (*P* < 0.001) (Figure 2).

The article "The Immunomodulatory Effects of Nidus Vespae on Human Peripheral Blood Immune Cells In Vitro" was published in 2015. Journal: Evid Based Complement Alternat Med.

### 3.3. Tumor Cell-Killing Activity of CTL

As shown in Figure 3, the cytotoxicity index of the CTL against SGC-7901 after treatment with NVD was 9.35%, 10.80%, and 10.25% for 10 : 1, 20 : 1, and 40 : 1, respectively, which were significantly greater than control (2.39%, 3.43%, and 3.28%, *P* < 0.01). No significant differences were observed between NVD treated CTL at different effector/target ratios and the untreated controls.

### 3.4. Effect of NVD on IgG Production

As shown in Figure 4, NVD significantly increased the IgG antibody production of resting B lymphocytes, as compared with the control group (*P* < 0.001, *P* < 0.001, and *P* < 0.05 for 5000, 2500, and 250 *μ*g/mL, resp.).

### 3.5. TNF-*α* and IL-6 Secretions of Monocytes

The TNF-*α* and IL-6 levels in each supernatant were quantitated by ELISA and analyzed by one-way ANOVA. The results were shown in Figure 5. The TNF-*α* and IL-6 secretions of monocytes were increased markedly when the NVD concentration was 5000 and 2500 *μ*g/mL, as compared with the control groups (*P* < 0.0001). When the reaction concentration was 250 *μ*g/mL, there were no significant secretions of TNF-*α* and IL-6.

### 3.6. Tumor Cell Phagocytosis of Monocytes

As shown in Figure 6, there was no significant effect of NVD on monocytes proliferation, nor on tumor cells inhibition. However, there was a marked decrease of OD values in the monocytes + NVD + SGC-7901 group, as compared with the monocytes + SGC-7901 group (*P* < 0.0001). It indicated that NVD significantly promoted the phagocytosis of monocytes on tumor cells.

## 4. Discussion

Most of the present studies about bee products were focused on propolis and honey. Numbers of experimental works revealed that propolis and jungle honey possess potent antitumor activity [7, 15–17]. However, the existing studies about Nidus Vespae were only confined to the oral diseases [18–20], and few studies were carried out to investigate the potential mechanisms by which Nidus Vespae exerts antitumor effects. Therefore, the main purpose of this paper was to investigate the immunomodulatory effects of Nidus Vespae on human peripheral blood immune cells* in vitro*, in order to explore the potential mechanisms of NVD in antitumor therapy.

The article "The Immunomodulatory Effects of Nidus Vespae on Human Peripheral Blood Immune Cells In Vitro" was published in 2015. Journal: Evid Based Complement Alternat Med.

Some kinds of Chinese herbs were found to be able to suppress tumor cells proliferation, thus exerting their antitumor effects [4]. In this study, instead, the viability of gastric cells SGC-7901, HGC-27, and NCI-N87 exhibited no significant differences among different concentration levels of Nidus Vespae (Figure 1). It indicates that NVD does not lead to the SGC-7901, HGC-27, and NCI-N87 toxicities in the studied concentrations. Accordingly, there must be other mechanisms involved in the antitumor activity of NVD. For instance, the mechanisms may be related to immune regulation, induction of tumor cell apoptosis, antiangiogenesis, inhibition of telomerase activity, and so on. In this study, we focused our attention on the regulation activity of NVD on human peripheral blood immune cells of gastric cancer patients.

Tumor immunotherapy requires proper manipulation of the immune system to identify and destroy the tumor cells as nonself. For this reason, we investigated the stimulation effect of NVD on proliferation of PBMC isolated from gastric cancer patients. The result showed that NVD could significantly promote the PBMC proliferation in a time- and concentration-dependent manner (Figure 2). Lymphocyte is the main component of PBMC, which primarily consisted of T and B cells. Although we did not separate T and B cells from PBMC to investigate their respective functions, the results showed that NVD could induce tumor-associated antigen-specific cytotoxic T cell response from PBMC (Figure 3) and promote IgG secretion of B cells (Figure 4), thus suggesting its immunostimulatory action toward T and B cells. However, two questions remain: Is the induction of CTL response against tumor cells simply due to the promotion of CTL proliferation or also through the enhancement of CTL killing efficiency? Is the promotion of IgG production of B cells due to the direct effects of NVD on B cells, or also through indirect effects of inducing Th2 cell to produce IL-4, IL-5, IL-6, and so forth and then stimulate the B cell to produce antibodies? These questions merit further studies and explorations.

It has been demonstrated that function of monocyte could be regulated by numbers of different Chinese herbs [15]. We investigated the antitumor activity of NVD by testing the response of monocytes. The results showed that TNF-*α* and IL-6 productions by monocytes incubated with NVD at different concentration levels (5000 and 2500 *μ*g/mL) increased* in vitro* (Figure 5), but the proliferation activity of monocytes and tumor cell toxicity did not seem to be affected by NVD. However, the phagocytosis of monocytes was significantly improved when treated with NVD (Figure 6). These results indicated that NVD may be partially involved in tumor immunoregulation, and the effect may depend on the enhancing of immune cells response, rather than the inhibition of tumor cells activity. Similar findings were previously reported in* Astragalus membranaceus* extract [21] and propolis [15].

The article "The Immunomodulatory Effects of Nidus Vespae on Human Peripheral Blood Immune Cells In Vitro" was published in 2015. Journal: Evid Based Complement Alternat Med.

In conclusion, the Nidus Vespae decoction could promote the proliferation of human PBMC, enhance the tumor cell-killing activity of CTL, elevate the IgG production of B cells, and strengthen the tumor cell phagocytosis as well as the cytokines (TNF-*α* and IL-6) production of monocytes. These results provide some possible scientific basis for the clinical application of Nidus Vespae decoction in traditional Chinese medicine. We believe that it may open the door for further studies on its use in tumor immunotherapy.

## Figures and Tables

**Figure 1:** Cell viability (%) of tumor cell lines after incubation with Nidus Vespae (10, 100, 1000, 2500, 5000, and 10000 *μ*g/mL) or control for 24 h. Data were analyzed by one-way ANOVA and presented as mean and standard deviation. No significant differences were observed between all concentrations; yet it showed increased tendencies of viability.

**Figure 2:** Proliferation rate (%) of PBMC after incubation with Nidus Vespae (75, 150, 300, 600, 1250, 2500, and 5000 *μ*g/mL), control, or ConA (5 *μ*g/mL) for 24 h, 48 h, or 72 h. Data were analyzed by two-way ANOVA and presented as mean and standard deviation (*n* = 5). It showed that NVD significantly promotes the proliferation of PBMC in a concentration- and time-dependent manner.  ^*∗*^Significantly different from PBS control groups (*P* < 0.001).

**Figure 3:** ^51^Cr releasing assay of CTL cytotoxicity against SGC-7901 target cells. CTL cytotoxicity was compared between NVD treated CTL (■) and untreated controls (○) (*n* = 10). Comparisons were statistically significant as compared with untreated controls (*P* < 0.01). No significant differences were observed between different effector/target ratios. Data were analysed by two-way ANOVA and presented as mean and standard deviation.

**Figure 4:** IgG production (ng/mL) by resting B lymphocytes after incubation with Nidus Vespae (250, 2500, and 5000 *μ*g/mL), control, or 0.05% SAC for 24 h. Data were analyzed by one-way ANOVA and presented as mean and standard deviation (*n* = 10). Comparisons were statistically significant as compared with control.  ^*∗*^Significantly different from control group (*P* < 0.05),  ^*∗∗*^significantly different from control group (*P* < 0.001).

The article "The Immunomodulatory Effects of Nidus Vespae on Human Peripheral Blood Immune Cells In Vitro" was published in 2015. Journal: Evid Based Complement Alternat Med.

**Figure 5:** TNF-*α* and IL-6 secretion (pg/mL) by monocytes incubated with Nidus Vespae (250, 2500, and 5000 *μ*g/mL), control, or LPS (5 *μ*g/mL) for 24 h. Comparisons were statistically significant as compared with control. Data were analyzed by one-way ANOVA and presented as mean and standard deviation (*n* = 10).  ^*∗*^Significantly different from control group (*P* < 0.0001).

**Figure 6:** Effects of NVD on monocytes proliferation, tumor cells inhibition, and phagocytosis of monocytes. The monocytes phagocytosis of monocytes + NVD + SGC-7901 group was significantly stronger than that of monocytes + SGC-7901 group, and there were no significant effects of NVD on monocytes proliferation nor on tumor cells inhibition. Data were presented as mean and standard deviation (*n* = 10).  ^*∗*^Significantly different from monocytes + SGC-7901 group (*P* < 0.0001).
